This article has been retracted.

# Consistency analysis of microRNA‐arm expression reveals microRNA‐369‐5p/3p as tumor suppressors in gastric cancer

**DOI:** 10.1002/1878-0261.12527

**Published:** 2019-06-17

**Authors:** Lei Dong, Zhengyi Zhang, Jiayue Xu, Fang Wang, Yanni Ma, Feng Li, Chao Shen, Ziwen Liu, Junwu Zhang, Changzheng Liu, Ping Yi, Jia Yu

**Affiliations:** ^1^ Department of Biochemistry and Molecular Biology, Institute of Basic Medical Sciences Chinese Academy of Medical Sciences, School of Basic Medicine Peking Union Medical College Beijing China; ^2^ Department of General Surgery, Peking Union Medical College Hospital Chinese Academy of Medical Sciences, Peking Union Medical College Beijing China; ^3^ NHC Key Laboratory of Systems Biology of Pathogens and Christophe Mérieux Laboratory, IPB, CAMS‐Fondation Mérieux, Institute of Pathogen Biology (IPB) Chinese Academy of Medical Sciences (CAMS) & Peking Union Medical College Beijing China; ^4^ Department of Obstetrics and Gynecology The Third Affiliated Hospital of Chongqing Medical University Chongqing China

**Keywords:** AKT1, c‐Jun, DNA methylation, gastric cancer, microRNA

## Abstract

The 5p and 3p arms of microRNA (miRNA) are typically generated from the same precursor, and one arm influences protein output, while the other has a short half‐life. However, a few miR‐5p/3p pairs have been reported to co‐exist in cancer cells. Here, we performed a genome‐wide analysis of miRNA expression in gastric cancer (GC) cells to systematically investigate the co‐expression profile of miR‐5p/3p in gastric tumorigenesis. We discovered that only 41 miR‐5p/3p pairs out of 1749 analyzed miRNA were co‐expressed. Specifically, abnormal expression of miR‐369‐5p and miR‐369‐3p was correlated with GC progression. Importantly, both *in vitro* and *in vivo* assays revealed that miR‐369‐5p and miR‐369‐3p exhibited tumor‐suppressive roles by regulating jun proto‐oncogene and v‐akt murine thymoma viral oncogene homolog 1 function in GC cells, respectively. Moreover, we observed that miR‐369 was inactivated in GC tissues due to DNA methylation. We also showed that inhibition of miR‐369‐5p/3p attenuated the effect of azacitidine (AZA) treatment on suppressing cell growth and invasion. These results suggest that the therapeutic efficacy of AZA in GC is at least partly attributable to miR‐369 activation. Overall, our findings provide convincing evidence that both the 5p and 3p arms of miRNA co‐expressed in GC and DNA methylation‐induced miR‐369 signaling contribute to GC progression.

**Abbreviations**
AKT1: v‐akt murine thymoma viral oncogene homolog 1
AML/MDS: acute myeloid leukemias and myelodysplastic syndrome
AZA: azacitidine
BSP: bisulfite sequencing
CCK‐8: cell counting kit‐8
c‐Jun: jun proto‐oncogene
FDA: U.S. Food and Drug Administration
GC: gastric cancer
H&E: hematoxylin and eosin
HOXA1: homeobox A1
HOXA11: homeobox A11
IP: immunoprecipitation
MeDIP: methylated DNA immunoprecipitation
miRNA: microRNA
MLH1: mutL homolog 1
MUC4: mucin 4, cell surface associated
qRT‐PCR: quantitative real-time PCR
RISC: RNA‐induced silencing complex
ROCK1: Rho associated coiled‐coil‐containing protein kinase 1
RUNX3: RUNX family transcription factor 3
Scr: scramble
TIAM1: T cell lymphoma invasion and metastasis 1
TSA: trichostatin A

## 1 Introduction

The microRNA (miRNA) genes are transcribed into primary miRNA transcripts, called pri‐miRNA, and these pri‐miRNA undergo nuclear cleavage to liberate miRNA precursors (pre‐miRNA) (Bartel, 2004). Following nucleocytoplasmic export, pre‐miRNA are further processed to generate the 5p and 3p arms of miRNA (miR‐5p and miR‐3p), here denoted as miRNA pairs (Lee *et al.*, 2003; Lee *et al.*, 2002). In the canonical model of miRNA biogenesis, one of the two arms of miRNA affects the output of protein‐coding genes through incorporating into RNA‐induced silencing complex (RISC) and the other one is typically recognized as a bypass product (Bartel, 2004; Song *et al.*, 2003). Previous studies have clearly indicated that ectopic expression of miRNA can have an oncogenic or tumor‐suppressive effect on tumorigenesis and progression (Lin and Gregory, 2015). However, most of these studies only focus on one arm of the specific miRNA in diverse cancer types. Until recently, the roles of several miRNA pairs have been reported. For instance, the miR‐126‐5p/3p pair represses breast cancer metastasis via directly inhibiting chemokine (C‐X‐C motif) ligand 12, and the miR‐27a‐5p/3p pair contributes to osteosarcoma cell invasion by negatively regulating core‐binding factor, runt domain, alpha subunit 2; translocated to, 3 (Salah *et al.*, 2015; Zhang *et al.*, 2013). These findings suggest that one miRNA transcript can regulate each cellular process though two pathways mediated by either its 5p or 3p arm.

Cancer cells acquire new characteristics to overcome physiological homeostasis, and they ultimately become malignant through a multiple‐step process (Hanahan and Weinberg, 2011). Epigenetic modifications are common events in carcinogenesis, and various cancer hallmarks, including malignant self‐renewal, differentiation blockade, cell death resistance, evasion of immune destruction, and tissue metastasis, are profoundly affected by alterations in the epigenome, suggesting that abnormal epigenetic regulation directly influences the tumorigenesis and progression. Importantly, DNA methylation studies provided the first early evidence linking epigenetic modifications to cancer (Feinberg and Tycko, 2004). Although the initial data were simply correlative, they represented a possible association between epigenetic pathways and tumorigenesis (Dawson and Kouzarides, 2012; Yang *et al.*, 2014). Recent advances have indicated that DNA methylation contributed to the inactivation of numerous tumor suppressors, including protein‐coding genes and miRNA (Issa, 2004; Kristensen *et al.*, 2014). These findings suggested that miRNA‐induced signaling might be a potential therapeutic target of hypomethylating agents. Despite this progress, many questions remain unanswered. It is still unknown whether the concerted effect of miR‐5p and miR‐3p is a common event in tumorigenesis. The mechanism of miR‐5p/3p inactivation remains unclear. Moreover, the genetic determinant of specific miRNA pair needs to be further elucidated.

Herein, we performed a comprehensive analysis of miRNA expression in gastric cancer (GC) using The Cancer Genome Atlas (TCGA) dataset and identified five deregulated miRNA pairs. Of them, miR‐369‐5p and miR‐369‐3p were simultaneously suppressed in GC samples due to DNA methylation. Moreover, we show that miR‐369‐5p/3p pair‐induced jun proto‐oncogene (c‐Jun)/AKT oncogenic signaling might be a potential therapeutic target of azacitidine (AZA).

## 2 Materials and methods

### 2.1 Patient dataset and clinical specimens

A total of 424 patients with GC and their related clinical information were obtained from TCGA data portal (https://www.cancer.gov/about-nci/organization/ccg/research/structural-genomics/tcga). A total of 107 fresh GC samples obtained from Peking Union Medical College hospital and Daping hospital were included in this study. Tissues were immediately snap‐frozen in liquid nitrogen after resection and stored at −80 °C. The study was approved by the ethical board of hospitals and the ethical board of the Institute of Basic Medical Sciences, Chinese Academy of Medical Sciences. The study methodologies conformed to the standards set by the Declaration of Helsinki, and patients signed the informed consent prior to sample collection. All of the samples were histologically confirmed by staining with hematoxylin–eosin (H&E). The patient characteristic data are provided in Tables S1 and S2.

### 2.2 Cell culture and drug treatment

The normal gastric epithelial cell line (GES‐1) was a kind gift from J. Shi. HEK293T, and the GC cell lines, HGC27, SGC7091, MGC803, and MKN45 cell lines were obtained from the American Type Culture Collection (ATCC, Manassas, Virginia, USA) and grown in Dulbecco’s modified Eagle’s medium with 10% FBS (Hyclone; General Electric Company, Boston, USA) at 37 °C in a 5% CO_2_ cell culture incubator. Cell lines were tested 1 month prior to the experiments by morphological evaluation under the microscope, growth curve analysis, and detection of mycoplasma levels according to the ATCC cell line verification test recommendations. GC cells were seeded overnight and then treated with 5 μm AZA (Sigma‐Aldrich, St. Louis, USA) for 72 h, 300 nm trichostatin A (TSA; Sigma‐Aldrich) for 24 h, or 5 μm AZA alone or in combination with TSA for 48 h. The harvested cells were used for DNA and RNA isolation.

### 2.3 Cumulative frequency analysis of the miR‐5p/3p ratio

To determine the inflexion point of miR‐5p/3p ratio, we use the following formula to calculate the ratio of miR‐5p and miR‐3p in GC tissues and the matched normal control tissues, respectively. Ratio = Log10 (miR‐5p/miR‐3p). Then, the cumulative frequency curve based on ratio of miR‐5p and miR‐3p is drawn as previously described (Erlandsson et al., 2017). The curve rising sharply until the infection point Ratio = 2, after that the curve tends to saturation.

### 2.4 Bisulfite modification and genomic sequencing

A bisulfite sequencing (BSP) assay was performed as previously described (Jacinto *et al.*, 2007). Bisulfite conversion was conducted using the MethylDetector Bisulfite Modification Kit (Active Motif, Carlsbad, USA) according to the manufacturer’s instructions. The fragments of interest were amplified using specific primers designed using MethPrimer software (Li *et al*. 2002) (Table S3). PCR products were gel purified and cloned into the pGEM‐T vector (Promega, Madison, USA). Individual bacterial colonies were selected to perform DNA sequencing.

### 2.5 Quantification of RNA and protein

Total RNA was extracted from cells and tissues using Trizol (Invitrogen, Carlsbad, CA, USA) according to the manufacturer′s instruction. A quantitative real‐time PCR (qRT‐PCR) assay was conducted to detect the miRNA and mRNA expression as previously described (Wang *et al.*, 2015). The primer sequences are available in Tables S4 and S5.

Western blot analysis of proteins was performed as previously described (Liu *et al.*, 2010). The antibodies included those against phosphorylated‐c‐Jun (p‐c‐Jun), c‐Jun, phosphorylated‐v‐akt murine thymoma viral oncogene homolog 1 (p‐AKT1), and AKT1 from Cell Signaling Technology Inc. (Danvers, USA) and GAPDH from Abcam (Cambridge, USA).

### 2.6 Constructs, reagents, and assays

The 3′UTR of the human AKT1 and c‐Jun mRNA was cloned in between the Not1 and Xba1 sites of pRL‐TK (Promega). Mutation of the AKT1 and c‐Jun sequence was created by using a QuickChange site‐directed mutagenesis kit (Stratagene, California, USA). Sequences of the primers are shown in Table S5. miRNA mimics and inhibitors specifying miR‐369‐5p/3p and control miRNA mimic/inhibitor were obtained from Dharmcon Inc. (Colorado, USA) AZA is a product of Sigma Ltd.

293T cells were seeded onto 24‐well plates (1 × 10^5^ cells per well) the day before transfections were performed, and the detection of the activity of reporter gene was performed as previously described (Wang *et al.*, 2015).

### 2.7 Cell proliferation, migration, and invasion assays

The cell growth was assessed using cell counting kit‐8 (CCK‐8; DOJINDO LABORATORIES, Kumamoto, Japan) and apoptosis assay as previously described (Liu *et al.*, 2010). Scratch wound assay was conducted to detect cell migration and performed as described (Yu *et al.*, 2010). Invasion assay was evaluated by the ability of cells passing through Matrigel‐coated membrane matrix (BD Biosciences, San Jose, USA) and performed as described (Liu *et al.*, 2010).

### 2.8 Immunohistochemistry

Immunohistochemistry (IHC) was performed to assess the levels of Ki‐67, caspase‐3, p‐c‐Jun, c‐Jun, p‐AKT1, and AKT1 as previously described (Liu *et al.*, 2010). IHC staining was evaluated as previously described (Waltregny et al., 1998).

### 2.9 Tumorigenicity and metastasis formation assays

All of the experimental procedures involving animals were performed in accordance with the Guide for the Care and Use of Laboratory Animals (NIH publications Nos. 80–23, revised 1996) and according to the institutional ethical guidelines of Peking Union Medical College for animal experiments. Tumorigenicity and metastasis formation assay were performed as described (Du *et al.*, 2017; Liang *et al.*, 2013).

### 2.10 Statistical analysis

Each experiment was repeated at least three times. Student's *t*‐test (two‐tailed) was performed to compare two groups (*P* < 0.05 was considered significant) unless otherwise indicated (χ^2^ test), and three‐group data were analyzed using one‐way analysis of variance. Correlations between miRNA expression and clinicopathological features were analyzed using nonparametric tests such as the Mann–Whitney *U*‐test for differences between two groups and the Kruskal–Wallis test for differences between three and more groups. All statistical analyses were performed using spss 16.0 software (SPSS Inc., Chicago, IL, USA). *P* values < 0.05 were considered statistically significant.

## 3 Results

### 3.1 Co‐expression analysis of miR‐5p/3p in GC tissues

Previous studies have reported that co‐expression of specific miRNA pairs in diverse cancer cells (Salah *et al.*, 2015; Zhang *et al.*, 2013). Here, we performed a comprehensive analysis of miR‐5p and miR‐3p expression in GC tissues using the entire TCGA GC cohort (424 patients). The workflow for differential expression analysis of miRNA is depicted in Fig. 1A. A total of 1749 miRNA were included in this analysis and we found that the expression of 126 miR‐5ps and 151 miR‐3ps was suppressed, while the expression of 45 miR‐5ps and 31 miR‐3ps was induced (Fig. 1B,1). Among these, 41 miRNA pairs had comparable expression profiles (30 were downregulated and 11 were upregulated; Fig. 1D; Table S6 and S7). Overall, the miR‐5p and miR‐3p with high enrichment typically show higher tendency of functional collaboration. We thus examined the ratio of miR‐5p/miR‐3p in both GC and matched normal tissues. An inflexion point on the cumulative rate curve (5p/3p = 100) was observed, and we identified 20 miRNA under this threshold (Fig. 1E, 1; Table S8), which suggests that only a small number of miRNA (20/1749) might be directly linked to regulatory function in gastric tumorigenesis (Fig. 1G). More interestingly, these data are similar to results reported by Lim and coworkers, who showed ~ 100‐fold difference in cloning frequency of miR‐5p and miR‐3p in *Caenorhabditis elegans* genome (Lim *et al.*, 2003). To further narrow down the candidate miRNA pairs with potential co‐regulatory roles, we decreased the ratio cutoff of miR‐5p and miR‐3p from 100 to 2, so that the ratio of miR‐5p/3p was smaller than a twofold difference in at least one of the two sample types (GC tissues and matched normal control tissues). New analysis identified 5 miR‐5p/3p miRNA pairs of which three were downregulated and two were upregulated, accounting for a very small percent of the total examined miRNA (5/1749, 0.29%; Fig. 1H,I).

**Figure 1:** Expression Profiling of miRNA pairs in GC tissues. (A) Workflow for differential expression analysis of miRNA pairs in GC tissues. (B) The expression of miR‐5p and miR‐3p in the normal gastric and GC tissues from TCGA GC dataset. (C, D) Deregulated expression profiles of miR‐5p and miR‐3p are depicted as volcano plots with 126 miR‐5ps and 151 miR‐3ps downregulated (C). Of those, the 5p and 3p arms of 41 miRNA exhibited the same expression trends as shown in panel D (Down, 30; Up, 11). (E–G) The cumulative percentage analysis of miR‐5p/miR‐3p ratio showed an inflection point (Log5p/3p = 2.0) indicated with red arrows (E). The miR‐5p/miR‐3p ratio of 20 miRNA (Down, 12; Up, 8) was lower than a 100‐fold difference (F), representing ~ 2.3% of the examined 1749 miRNA (G). (H, I) The expression of five candidate miRNA pairs (Down, 3; Up, 2) was differentially regulated with an approximately twofold difference in enrichment of miR‐5p and miR‐3p in GC tissues.

Taken together, these data show that specific miRNA genes may undergo nonprevalent processing to generate two relatively stable miRNA arms.

### 3.2 Deregulated expression of miR‐369‐5p/3p pair was correlated with GC development

Since there are no reports documenting the function of miR‐369‐5p/3p, we specifically evaluated the role of miR‐369 pairs in GC cells. The expression of miR‐369‐5p/3p pair was examined in 107 paired GC tissues, which revealed that miR‐369‐5p and miR‐369‐3p were markedly decreased compared with the matched normal gastric tissues (miR‐369‐5p, 57/107; miR‐369‐3p, 49/107; Fig. 2A,2; Fig. S1). To determine whether the miR‐369 pair has a role in GC pathogenesis, we performed statistical correlation analysis between deregulated miR‐369‐5p/3p expression and GC progression in the examined tissues. Corresponding data of 105 patients with GC with detailed clinical information were included. Specifically, we observed that the expression of miR‐369 pair was negatively linked with the development of GC (Fig. 2C; Table S1). For instance, GC patients with low expression levels of miR‐369‐5p and miR‐369‐3p in tumors tended to have more extensive nodal involvement and low expression of this miRNA pair was significantly correlated with a more aggressive tumor phenotype (Fig. 2D,2).

**Figure 2:** Decreased expression of miR‐369‐5p/3p pair is linked to GC progression. (A, B) The qRT‐PCR analysis revealed decreased levels of miR‐369‐5p (A) and miR‐369‐3p (B) in the examined GC tissues (miR‐369‐5p, 53.2%; miR‐369‐3p, 45.8%). (C) Heatmap shows the correlation of miR‐369‐5p/‐3p expression with clinical pathological characteristics of GC patients. Each color‐coded cell represents the relative expression of miR‐369‐5p/3p and the characteristics of a particular patient. C indicates GC samples and N indicated the matched normal control. (D) The deregulated expression of miR‐369‐5p and miR‐369‐3p was linked with lymphatic invasion. (E) The expression of miR‐369‐5p and miR‐369‐3p was associated with pTNM stages.

Taken together, these data suggest that the miR‐369‐5p/3p pair is suppressed in gastric carcinogenesis and might act as a potential tumor suppressor in GC cells.

### 3.3 Overexpression of miR‐369‐5p or miR‐369‐3p suppresses GC cell growth

Next, we further investigated the function of miR‐369‐5p or miR‐369‐3p in GC cells. First, the expression of the miR‐369‐5p/3p pair was evaluated in several GC cells by the qRT‐PCR analysis (Fig. S2). Afterward, we conducted a short‐term transient transfection of miR‐369‐5p and miR‐369‐3p in MGC803 and HGC27 cells, which express low levels of miR‐369 (Fig. S3). Cell growth analysis revealed that miR‐369‐5p or miR‐369‐3p overexpression significantly lowered cell proliferation in GC cells (Fig. 3A). Assessment of apoptosis also suggested that overexpression of miR‐369‐5p or miR‐369‐3p led to an increase in early apoptotic cells (Fig. 3B). These data suggest a tumor‐suppressive role of the miR‐369‐5p/3p pair in GC cells.

**Figure 3:** Overexpression of miR‐369‐5p/3p inhibits GC cell growth. (A) miR‐369‐5p and miR‐369‐3p were overexpressed, and a CCK‐8 assay was conducted to determine the cell growth of MGC803 and HGC27 cells in 24‐h intervals up to 96 h. The overexpression of miR‐369‐5p and miR‐369‐3p led to the inhibition of GC cell growth. (B) An apoptosis assay was employed to determine the programmed cell death in MGC803 and HGC27 cells with miR‐369‐5p and miR‐369‐3p overexpression. Normalization of the percentage of early apoptotic cells is shown on the right. (C) Introduction of miR‐369‐5p and miR‐369‐3p dampened the capacity of GC tumor formation *in vivo* as shown by xenograft models. Images of the representative nude mice from each group (*n* = 5/group) are displayed on the left. The graph represents the tumor volumes at the indicated days during the experiment for the following three groups: Scr‐, miR‐369‐5p‐, and miR‐369‐3p‐treated MGC803 cells (right panel). (D) Images of the removed tumors from nude mice are shown (left panel). The tumor weights are shown on the right. (E–H) Pathological analysis of tissue sections from recipient mice including H&E staining (E) and labeling with anti‐Ki‐67 and anti‐caspase‐3 (F–H) was performed at 4 weeks postinjection. The expression of Ki‐67 and caspase‐3 in the tissue sections was normalized to the Scr group (right panel). Scale bars: 100 μm (H&E) and 20 μm (IHC). Average values and SDs were calculated from triplicate samples. *P* values were based on Student's *t*‐test unless otherwise indicated. *P < 0.05, **P < 0.01, ***P < 0.001.

Next, we examined the role of the miR‐369‐5p/3p pair *in vivo*. To this end, we subcutaneously transplanted MGC803 cells with miR‐369‐5p or miR‐369‐3p overexpression into the posterior flanks of immunodeficient nude mice. After 4 weeks, we observed that miR‐369‐5p and miR‐369‐3p inhibited the growth of MGC803‐engrafted tumors compared to control‐treated tumors treated with scramble (Scr) sequence evidenced by tumor volumes evaluation (Fig. 3C). Significantly smaller tumor weights were found in mice treated with miR‐369‐5p or miR‐369‐3p compared to the Scr control group (Fig. 3D). Moreover, the expression of Ki‐67 and caspase‐3 was immunohistochemically detected in randomly selected xenograft mouse tumors, revealing that the miR‐369‐5p/3p pair suppressed the growth of GC cells (Fig. 3E–H).

Taken together, these data indicate that overexpression of miR‐369 pair remarkably inhibits the tumorigenicity of GC cells *in vitro* and *in vivo*.

### 3.4 Overexpression of miR‐369‐5p/3p pair decreases GC cell movement

The roles of miR‐369‐5p and miR‐369‐3p in GC cell migration and invasion were further investigated to assess their role in GC metastasis. To test this aim, we performed wound‐healing assays in MGC803 and HGC27 cells which overexpressed miR‐369‐5p and miR‐369‐3p in MGC803 and HGC27 cells to determine GC cell migration. We found that MGC803 cells treated with miR‐369‐5p or miR‐369‐3p sealed only ~ 65% of the wound area after 36 h compared to MGC803 cells treated with Scr sequence (Fig. 4A). Similar results were observed in HGC27 cells (Fig. 4B). Furthermore, *in vitro* transwell assays were conducted to evaluate the effect of the miR‐369‐5p/3p pair on GC cell movement, which indicated that the miR‐369 pair markedly inhibited cell migration in MGC803 and HGC27 cells (Fig. 4C). Next, we conducted an *in vitro* invasion assay and observed that miR‐369‐5p and miR‐369‐3p overexpression significantly decreased the invasion of MGC803 and HGC27 cells compared to cells given Scr treatment (Fig. 4D). The *in vivo* metastasis assays were used to further confirm the *in vitro* findings. For the *in vivo* metastasis assays, 5 × 10^5^ live MGC803 cells were resuspended in 0.1 mL of phosphate‐buffered saline after infection with Lenti‐369‐5p, Lenti‐369‐3p, or Lenti‐scr. Next, the infected cells were injected into the lateral tail veins of nude mice, and 7 weeks after injection, the animals were sacrificed, and the lungs and livers were collected for histology. We observed that the number of hepatic metastases in mice that were injected with Lenti‐369‐5p/3p‐infected MGC803 cells was significantly lower compared to mice injected with Lenti‐scr‐infected cells (Fig. 4E,4). Histopathological assessment of liver tissues by H&E staining identified more metastatic nodules in Lenti‐scr‐treated mice compared to Lenti‐369‐5p/3p‐infected mice (Fig. 4G,H). Similar results were observed in the lung tissues although no significant changes were observed in the gross examination (Fig. 4I,J).

**Figure 4:** Overexpression of miR‐369‐5p/3p suppresses GC cell invasion. (A, B) The wound‐healing assay was performed with miR‐369‐5p/3p mimics or Scr transfection in MGC803 (A) and HGC27 (B) cell, phase‐contrast photographs were every 12 h, and AxioVision software was used to temporally assess the wound closure percentage from typical representatives (*n* = 3). Scale bars: 500 μm. (C, D)* in vitro* transwell assay (C) and *in vitro* invasion assay (D) were performed in MGC803 and HGC27 cells upon transfection with miR‐369‐5p/3p mimics or Scr. Representative photographs are shown (magnification: 200×). Scale bars: 50 μm. The migrated or invasive cells were normalized as shown (right). (E, F) MGC803 cells infected with Lenti‐369‐5p, Lenti‐369‐3p, or Lenti‐scr were injected into nude mice through the lateral tail vein. The mice were sacrificed at 5 weeks postinjection (E). The circles indicate the metastases. The gross assessment of the dissected livers was performed (F). (G–J) Histological analysis was performed on sections of the livers (G, H) and lungs (I, J) from the mice that were injected with Lenti‐scr‐ or Lenti‐369‐5p/3p‐infected MGC803 cells. Magnified images are shown within the boxed regions. Scale bars: 50 μm. The calculated number of metastatic nodes in the liver and lung is shown. Average values and SDs were calculated from triplicate samples. *P* values were based on Student's *t*‐test unless otherwise indicated. **P < 0.01, ***P < 0.001.

Altogether, these findings suggest that miR‐369‐5p and miR‐369‐3p suppress GC cell invasion and metastasis.

### 3.5 miR‐369‐5p targets endogenous c‐Jun

To identify the mRNA targets of miR‐369‐5p relevant to gastric tumorigenesis, we used the miRanda miRNA target prediction program, which suggested that c‐Jun was a potential target of miR‐369‐5p. The 3´UTR of *c‐Jun* houses a sequence that matches the 7‐mer seed sequence contained within the sequence of miR‐369‐5p (Fig. 5A). Transfection of the *c‐Jun*‐3´UTR‐luciferase reporter in combination with the miR‐369‐5p mimic was conducted in 293T cells and showed that miR‐369‐5p inhibited the luciferase activity. Importantly, mutation of the miR‐369‐5p sites abrogated this inhibition (Fig. 5B). Furthermore, increased levels of miR‐369‐5p in MGC803 and HGC27 cells led to decreased protein levels of c‐Jun (Fig. 5C).

**Figure 5:** miR‐369‐5p and 369‐3p target endogenous c‐Jun and AKT1 in GC. (A) Sequences within the 3′‐UTR of *c‐Jun* and *AKT1* were targeted by miR‐369‐5p and miR‐369‐3p, respectively, and those shaded in gray represent mutants of the miR‐369‐matched seed sequence. (B) The luciferase activity was reduced when miR‐369‐5p was bound to the segment containing the target sequence within the 3′‐UTR in *c‐Jun* mRNA, while miR‐369‐5p‐dependent repression was abolished upon mutation of the seed sequence. (C) Immunoblotting analysis was performed to assess the protein level of c‐Jun in HGC27 and MGC803 cells upon miR‐369‐5p mimic treatment. (D) The protein levels of c‐Jun and p‐c‐Jun were increased in the GC tissues compared to the matched normal tissues. The expression of c‐Jun and p‐c‐Jun in the tissue sections was normalized as shown. (E) Representative images of c‐Jun and p‐c‐Jun IHC analysis in GC samples. Normalization of the protein expression is shown compared to the matched normal control. (F) The luciferase activity was decreased when miR‐369‐3p was bound to the segment containing the target sequence within the 3′‐UTR in *AKT1* mRNA, while miR‐369‐3p‐dependent repression was abolished by mutating the seed sequence. (G) Immunoblotting analysis indicated the miR‐369‐3p overexpression resulted in a diminished AKT1 protein levels in MGC803 and HGC27 cells and the normalized expression of AKT1 protein to Scr‐treated GC cells is shown below the panels. (H) The protein levels of AKT1 and p‐AKT1 were increased in the GC tissues compared to the matched normal tissues. The expression of c‐Jun and p‐c‐Jun in the tissue sections was normalized as shown. (I) Representative images of AKT1 and p‐AKT1 IHC analysis in GC samples. The normalized expression levels of AKT1 and p‐AKT1 are shown compared to the matched normal control. For all immunoblots, GAPDH was used as a loading control and the numbers below the panels represent the normalized protein expression levels. For histology and IHC panels, magnification is 20× and scale bars are 50 μm. Average values and SDs were calculated from triplicate samples. *P* values were based on Student's *t*‐test unless otherwise indicated. *P < 0.05, **P < 0.01.

Next, we examined the expression of c‐Jun in GC tissues with downregulated expression of miR‐369‐5p. Western blot analysis of eight pairs of GC tissues with decreased levels of miR‐369‐5p (Fig. S4A) demonstrated that the levels of c‐Jun were increased in these tissues (Fig. 5D). Immunohistochemical analysis also indicated that c‐Jun expression was increased in GC tissues compared to adjacent normal gastric tissues (Fig. 5E; Fig. 4B).

Altogether, these data suggest that c‐Jun is a direct target regulated by miR‐369‐5p in GC cells.

### 3.6 AKT1 is a direct target of miR‐369‐3p

Computation analysis using miRanda miRNA target prediction identified human AKT1 as a potential target of miR‐369‐3p in two regions within its 3′UTR (Fig. 5A). To validate this finding, we constructed a reporter plasmid to include the predicted miR‐369‐3p target sequence within the AKT1 3′UTR region, and then, we co‐transfected this reporter plasmid with either Scr or miR‐369‐3p mimic into 293T cells. The luciferase assay indicated a significant decrease in the luciferase activity. Mutation of the target sites in miR‐369‐3p at positions 1 and/or 2 completely abrogated this inhibition in luciferase activity, indicating the specificity of the interaction between miR‐369‐3p and its target regions (Fig. 5F). Western blot analysis further confirmed that miR‐369‐3p overexpression was associated with reduced levels of AKT1 protein compared to control (Fig. 5G).

Next, we examined the link between miR‐369‐3p and AKT1 in eight pairs of GC tissues. Analysis by qRT‐PCR revealed that miR‐369‐3p was significantly reduced in GC samples compared to the matched normal gastric tissues (Fig. S4C). Further immunoblots indicated that the protein levels of AKT1 were decreased in these examined GC tissues (Fig. 5H). Similar results were observed in the immunohistochemical assessment (Fig. 5I; Fig. S4D).

Taken together, our data support the finding that miR‐369‐3p directly targets AKT1 in GC cells.

### 3.7 DNA methylation reduces the expression of the miR‐369‐5p/3p pair

We observed decreased expression of miR‐369‐5p and miR‐369‐3p in GC cells and wanted to determine whether the inactivation of miR‐369‐5p/3p pair was due to epigenetic modifications. To this end, we treated GC cells with TSA and 5‐azacytidine (AZA). Gene expression analysis by qRT‐PCR revealed that both miR‐369‐5p and miR‐369‐3p were increased by TSA or AZA treatment in GC cells (Fig. 6A), suggesting that DNA methylation‐induced miR‐369 suppression might be a frequent event in gastric tumorigenesis. In order to validate this hypothesis, the methylation status of the *miR‐369* promoter was evaluated by BSP sequencing. We analyzed the potential CpG islands located within the *miR‐369* promoter (Fig. 6B) and employed a BSP assay in 20 cases of GC tissues. Meanwhile, qRT‐PCR analysis was used to investigate the expression of primary miR‐369 (pri‐miR‐369) in these GC samples and revealed that suppression of pri‐miR‐369 in 12 cases and induction in five cases of GC (Fig. 6C). Association analysis between the BSP analysis and pri‐miR‐369 expression data revealed that DNA methylation was correlated with reduced levels of miR‐369 (Fig. 6D; Fig. S5).

**Figure 6:** DNA methylation deregulates the miR‐369‐5p/3p pair in GCs. (A) The expression of miR‐369‐5p and miR‐369‐3p was induced by AZA treatment in MGC803 and HGC27 cells as shown by qRT‐PCR analysis. Data were normalized to U6 snRNA. (B) Schematic representation of the potential hypermethylated sites located at the miR‐369 promoter. BSP PCR primers were designed using methprimer software, and a 300 nucleotide region containing 16 CpG islands was amplified after bisulfite conversion. (C) The qRT‐PCR analysis was conducted to quantify the expression of primary miR‐369 (pri‐miR‐369) in 20 cases of GC tissue samples, and GPDAH was included as a control. (D) Bisulfite genomic sequencing of the miR‐369 promoter in 20 cases of GC tissues. The indicated methylation percentage was calculated based on the status of sequenced CpG islands. The methylated and unmethylated CpG dinucleotides are displayed as black circles and open circles, respectively. (E) The expression of c‐Jun was suppressed in MGC803 and HGC27 cells after AZA treatment as shown by qRT‐PCR and immunoblotting analyses. (F) The expression of AKT1 was downregulated in MGC803 and HGC27 cells after AZA treatment as shown by qRT‐PCR and immunoblotting analyses. For immunoblots, GAPDH served as a loading control, and data were normalized to DMSO‐treated GC cells. Average values and SDs were calculated from triplicate samples. *P* values were based on Student's *t*‐test unless otherwise indicated. *P < 0.05, **P < 0.01, ***P < 0.001.

Azacytidine treatment led to increased expression of miR‐369‐5p and miR‐369‐3p in GC cells, suggesting that AZA might also lead to decreased expression of c‐Jun and AKT1 in GC cells. To test this hypothesis, we performed qRT‐PCR and western blot analyses to evaluate the expression of c‐Jun and AKT1 in MGC803 and HGC27 cells treated with AZA. We found that AZA treatment resulted in a significant decrease of c‐Jun mRNA and protein levels in both cell lines (Fig. 6E,6).

Altogether, these data suggested that DNA methylation likely contributes to inactivation of miR‐369‐5p/3p pair in GCs.

### 3.8 AZA suppresses GC growth via the miR‐369 pair‐induced signaling

To determine the effect of AZA on GC cell growth or invasion through the miR‐369‐5p/3p pair‐induced signaling, we conducted a series of rescue assays in GC cells, where miR‐369 inhibitors (anti‐369‐5p or anti‐369‐3p) were transfected into GC cells following AZA treatment to modulate the miR‐369‐mediated c‐Jun/AKT1 pathway. The qRT‐PCR analysis revealed that AZA treatment induced both miR‐369‐5p and miR‐369‐3p, which was decreased by anti‐369 treatment in MGC803 and HGC27 cells (Fig. 7A). Moreover, the c‐Jun and AKT1 protein level decreased upon AZA treatment and increased with anti‐369 transfection as shown by immunoblots (Fig. 7B). The apoptosis assay and *in vitro* invasion assay showed that AZA treatment significantly promoted cell apoptosis and inhibited cell movement. However, inhibition of miR‐369‐5p/3p dramatically compromised the effect of AZA treatment, leading to increased GC cell growth (Fig. 7C–F) and invasion (Fig. 7G–J).

**Figure 7:** AZA treatment suppresses growth and invasion of GC cells through regulation of the miR‐369‐5p/3p‐mediated axis. (A) The expression of miR‐369‐5p and miR‐369‐3p was evaluated in AZA‐treated GC cells with or without miR‐369‐5p or miR‐369‐3p inhibition. (B) The protein levels of c‐Jun and AKT1 were assessed in AZA‐treated MGC803 (left panel) and HGC27 (right panel) cells with or without miR‐369‐5p or miR‐369‐3p inhibition. (C, D, E, F) The rescue experiment was conducted in MGC803 (C) and HGC27 (D) cells, and the extent of apoptosis was measured. Panels E and F represent the percentage of early apoptotic cells. (G, H, I, J) The rescue experiment was conducted in MGC803 (G) and HGC27 (H) cells, and *in vitro* invasion assay was performed. Representative images are shown in panels G and H (Magnification: 200×). Scale bars: 50 μm. The ratio of invasive cells was normalized as shown (I, J). (K, L) A schematic representation of AZA mechanism of action demonstrating its suppressive benefit in GC therapy via regulation of miR‐369‐5p/3p‐induced signaling. Average values and SDs were calculated from triplicate samples. *P* values were based on Student's *t*‐test unless otherwise indicated. *P < 0.05, **P < 0.01, ***P < 0.001.

Altogether, these findings suggest that DNA methylation‐induced miR‐369‐5p/3p signaling alteration is mediating gastric carcinogenesis and that AZA likely has clinical benefits for GC therapy through modulating the miR‐369‐mediated axis (Fig. 7K,L).

## 4 Discussion

The miR‐5p:miR‐3p duplex, generated from Dicer, is generally short‐lived compared to the single miRNA strand. Although numerous miRNA* are cloned and validated, they are thought to be bypass products with unknown functions and only one of the arms is typically incorporated into the RISC complex to induce gene silencing (Bartel, 2004). However, recent studies clearly indicate that both arms of miRNA (miR‐5p and miR‐3p) can negatively regulate the expression of target genes and exert biological or pathological function, such as miR‐126‐5p/3p (in breast cancer cells) and miR‐27a‐5p/3p (in osteosarcoma cells) (Salah *et al.*, 2015; Zhang *et al.*, 2013). Given these findings, we still do not understand whether co‐expression of miR‐5p and miR‐3p is frequent in the development and progression of tumorigenesis. In this study, we performed a comprehensive expression analysis of miR‐5p/3p pairs using TCGA GC dataset and observed that only a minority of pre‐miRNA can maintain two mature miRNA (41/1749), suggesting that an approximate percentage in enrichment of miR‐5p and miR‐3p may be an essential point for their functional collaboration. To test this idea, we compared the ratio of miR‐5p/miR‐3p using a cumulative frequency analysis and found that an ~ 100‐fold difference in enrichment of miR‐5p and miR‐3p is the critical threshold. Next, we selected miR‐369 to conduct further analysis because miR‐369‐5p and miR‐369‐3p show very comparable enrichment. Additionally, miR‐369 has been found to be conserved in placental mammals, which is a result of gradual evolution (Awan *et al.*, 2017). We demonstrated that suppression of miR‐369‐5p/3p pair in GC tissues is linked with GC progression and the miR‐369‐5p/3p pair functions as tumor suppressors as shown by the *in vitro* and *in vivo* data. The miRNA target prediction revealed that miR‐369‐5p and miR‐369‐3p could negatively regulate many protein‐coding genes, identifying that 138 mRNA were the common targets of these two miRNA. Of these potential targets, c‐Jun and AKT1 oncogenes were validated as the functional effectors of miR‐369‐5p and miR‐369‐3p in GC cells, respectively. These data suggest that the miR‐369‐5p/3p pair might actively exert the tumor‐suppressive function in GC.

Disrupted epigenetic modifications are frequently observed in carcinogenesis. Therefore, epigenetic regulators have the potential to function as anticancer drugs in cancer therapy. AZA is a type of hypomethylating agent that exerts significant suppressive effects in cancer progression (Dawson and Kouzarides, 2012). Since inactivation of miR‐369‐5p/3p pair is due to DNA methylation as shown by the BSP assays, we determined whether miR‐369‐induced signaling is a therapeutic target of AZA in GC cells. The rescue assays demonstrated that inhibition of the miR‐369‐5p/3p pair resulted in a dampened inhibitory impact of AZA on GC cell growth and invasion. Moreover, we also observed that AZA treatment induced the alteration of miRNA‐mediated signaling in GC cells. Our data indicate that epigenetic regulators, such as AZA, will likely exert clinical efficacy in GC therapy, which is partly mediated through the miR‐369‐5p/3p‐induced c‐Jun/AKT1 signaling.

## 5 Conclusions

In summary, our findings provide a comprehensive assessment of miR‐5p/3p in GC and clearly indicate that only a few of miRNA pairs exhibit co‐expression profiles. In particular, we have identified an axis comprised of DNA methylation‐induced miR‐369‐5p/3p pair, AKT‐1 and c‐Jun, which likely contributes to gastric tumorigenesis and progression.

## Conflict of interest

The authors declare no conflict of interest.

## Author contributions

Study concept and design: LD, ZZ, CL, and JY. Acquisition of data: LD, ZZ, JX, FW, YM, FL, and PY. Analysis and interpretation of data: LD, ZZ, CS, ZL, and JY. Drafting of the manuscript: LD, ZZ, FW, JZ, and YP. Critical revision of the manuscript for important intellectual content: JZ, CL, and JY. Statistical analysis: LD, ZZ, FL, CS, ZL, and YP. Obtained funding: JY, CL, and ZL. Administrative, technical, or material support: FW, YM, and JZ. Study supervision: CL and JY.

## Supporting information


**Fig. S1**. The expression of the miR‐369 pair is determined in GC tissues.
**Fig. S2**. The expression of the miR‐369 pair in GC cells.
**Fig. S3**. Overexpression of the miR‐369 pair in MGC803 and HGC27 cells.
**Fig. S4**. Expression analysis of miR‐369 pair and their targets in GC tissues.
**Fig. S5**. BSP sequencing in 20 GC tissue samples.

**Table S1**. Comparison of miR‐369 pair expression levels with clinico‐pathological features in patients with primary GC.
**Table S2**. Characteristics of the 424 GC patients.
**Table S3**. miR‐369 BSP sequencing primers.
**Table S4**. Primers used for the construction of luciferase reporters, qRT‐PCR analyses of mRNAs, and primary miR‐369.
**Table S5** **.** Sequences of miRNAs and U6 snRNA primers.
**Table S6** **. **Downregulated miRNA pairs in GCs.
**Table S7** **.** Upregulated miRNA pairs in GCs.
**Table S8**. The Ratio of miR‐5p/miR‐3p in GCs and the matched normal control.
